The article "Exploring tranquility: Eastern and Western perspectives" was published in 2022. Journal: Front Psychol.

# Exploring tranquility: Eastern and Western perspectives

**DOI:** 10.3389/fpsyg.2022.931827

**Published:** 2022-08-01

**Authors:** Vincent Ringgaard Christoffersen, Borut Škodlar, Mads Gram Henriksen

**Affiliations:** ^1^Independent Researcher, Copenhagen, Denmark; ^2^Unit for Psychotherapy, University Psychiatric Clinic Ljubljana, Ljubljana, Slovenia; ^3^Department of Psychiatry, Medical Faculty, University of Ljubljana, Ljubljana, Slovenia; ^4^Department of Communication, Center for Subjectivity Research, University of Copenhagen, Copenhagen, Denmark; ^5^Mental Health Center Amager, Copenhagen University Hospital, Copenhagen, Denmark

**Keywords:** consciousness, stoicism, yoga, Buddhism, meditation, mysticism, absorption, detachment

## Abstract

Although tranquility is a fundamental aspect of human life, the experiential nature of tranquility remains elusive. Traditionally, many philosophical, religious, spiritual, or mystical traditions in East and West have strived to reach tranquil experiences and produced texts serving as manuals to reach them. Yet, no attempt has been made to compare experiences of tranquility and explore what they may have in common. The purpose of this theoretical study is to explore the experiential nature of tranquility. First, we present examples of what we consider some of the most central experiences of tranquility in Eastern and Western traditions. For the sake of simplicity, we sort these examples into four categories based on their experiential focus: the body, emotions, the mind, and mysticism. Second, we offer an exploratory account of tranquility, arguing that the different examples of tranquility seem to share certain experiential features. More specifically, we propose that the shared features pertain both to the content or quality of the tranquil experiences, which involves a sense of presence and inner peace, and to the structure of these experiences, which seems to involve some degree of detachment and absorption.

## Introduction

From time immemorial, human beings have longed and strived for tranquility. Testimonies of this are widespread in sacred, philosophical, and medical texts, literature, and art. Throughout history and across cultures, contemplative, philosophical, spiritual, religious, and mystical traditions have developed their own practices to reach certain experiences of tranquility. Still, the nature of the various experiences of tranquility, the very purpose of reaching them, and their interpretation vary substantially, depending on the traditions’ cultural or religious configurations. From the perspective of everyday life, tranquility is not unknown to us. Occasionally we all feel tranquil, and we thus have an intuitive grasp of what tranquility means. Asked to define it, though, it tends to slip through our fingers, and we struggle to qualify the experience. Indeed, there is something puzzling about the experience of tranquility. On the one hand, it seems like a trivial phenomenon that everyone already is familiar with. On the other hand, it appears to be a complex phenomenon, requiring dedicated and enduring practice to reach.

In many Eastern traditions and practices (e.g., the six Brahmanic or orthodox schools such as Yoga, the non-orthodox or Shramanic schools of Indian philosophy such as Buddhism, Chinese traditions such as Daoism, etc.), tranquility has been a key focus for several thousand years. A few examples may illustrate this point. The first example is the introductory and *key* sutra (aphorism) of the Yoga Sutras (YS) of Patanjali, which reads “Yoga (is) bringing to complete cessation the functional modifications of citta [the mind]” (Karambelkar, 2012).^1^ In other words, the very purpose of Yoga is to still the mind. Another example is a famous verse of the Bhagavad Gita: “To the disunited (one not established in the Self) does not belong wisdom, nor has he meditation. To the unmeditative there is no tranquility. To the peaceless how comes happiness?” (2.66; Yogananda, 2013, p. 313). Yet another example is from the Soto Zen master, Shunryu Suzuki, who elaborating on calmness in zazen (i.e., the seated meditative practice of Zen) states, “When you are doing zazen, you are within the complete calmness of your mind; you do not feel anything. You just sit. But the calmness of your sitting will encourage you in your everyday life” (Suzuki, 2020, pp. 112–113). Finally, the work of the late Thich Nhat Hanh, a world-renowned Vietnamese Buddhist monk, is a powerful example of a dedicated, lifelong commitment to tranquility and peace [see, e.g., Hanh (2005)].

In Greek and Roman philosophy, tranquility was considered central to happiness (*eudaimonia*) by skeptics (e.g., Pyrrho of Elis and Sextus Empiricus), epicureans (e.g., Epicurus and Lucretius), and stoics (e.g., Chrysippus, Seneca, Epictetus, and Marcus Aurelius). Tranquility was the core experiential aspect of notions such as *ataraxia*, *apatheia*, and *euthymia*, which were important notions in these philosophical schools. These notions all describe a calm state of mind in which one is not disturbed or overwhelmed by strong emotions or passions, impulses or wishes. The term tranquility comes from the Latin *tranquillitas* (from *tranquillus*, quiet, calm, still), which, as Striker pointed out, is the term Cicero and Seneca used to translate Democritus’ *euthymia—*although the meaning of *tranquilllitas* is, in fact, closer to that of *ataraxia* (Striker, 1990, p. 98). In a seminal book, Sorabji (2000) illuminated how Greek and Roman ideas on tranquility found their way into early Christian thought through the works of Evagrius Ponticus and St. Augustine—ideas that also appear in the hesychast (gr. *hesychia*, inner peace or silence) tradition of the Eastern Orthodox Church, collected in *Philokalia*, and in the work of Christian mystics such as Eckhart (2009).

In contemporary philosophy and psychology, tranquility is sometimes regarded as an aspect of mental well-being (Soysa et al., 2021), considered a mood by some (e.g., Gallegos, 2017; Kriegel, 2019) and an emotion by others (e.g., Ellsworth and Smith, 1988; Berenbaum et al., 2019). Tranquility has also become an important topic in the growing literature on mindfulness (Bishop et al., 2004; Coleman and Coleman, 2019), metacognition (e.g., Schraw and Moshman, 1995; Jankowski and Holas, 2014; Dorjee, 2016), and equanimity (e.g., Juneau et al., 2020; Analayo, 2021). For example, tranquility has here been described in the context of emotional calmness or in relation to a state of mind, where, e.g., thoughts or sensations are noticed entering and leaving the field of awareness without engaging with them. Jon Kabat-Zinn, the founder of the Mindfulness-Based Stress Reduction approach and an ambassador of mindfulness in the West, has emphasized that Western mindfulness is strongly inspired by traditional meditative practices found in Buddhism (Kabat-Zinn, 2011).

Collectively, these examples illustrate that tranquility is a central concept in key texts of Yoga, Buddhism, and Christianity, in classical and contemporary philosophy, and in current psychological research. Still, we suggest that the phenomenon of tranquility has not yet come into full focus: Is tranquility an emotion or a mood? Is it an emotionless state or a state in which one’s emotions are balanced? Is tranquility always related to happiness? Is a relaxed body, emotional calmness, or a peaceful state of mind a prerequisite for experiencing tranquility? Is tranquility an ephemeral or enduring experience? Is the tranquility at stake in mystical states like that found in non-mystical states, etc.? Is there only one kind of tranquility or are there many kinds of tranquility and, if so, what do they have in common? If we are to answer such questions, a more comprehensive grasp of the experiential nature of tranquility is needed. The question therefore remains: What is tranquility?

## Exploring tranquility

Despite a remarkably rich and multifaceted history of tranquility across traditions and cultures, no comprehensive attempt has to the best of our knowledge been made to compare and map different forms of tranquil experiences and explore what they may have in common. Such a comparative analysis faces many challenges, including an appreciation of the different practices that seek to cultivate tranquil experiences and of the different natures, roles, and interpretations of these experiences in their respective philosophical, spiritual, or religious traditions. With this article, we hope to provide one key piece of the puzzle of what tranquility is.

Initially, however, we want to emphasize that we are not offering an exhaustive historical mapping of all kinds of tranquil states nor offering a definitive account of tranquility. Instead, we first offer examples of what we take to be some of the most central experiences of tranquility in Eastern and Western traditions. For the sake of textual simplicity, we sort these examples into four categories based on their primary experiential focus: the body, emotions, the mind, and mysticism. While this categorization provides a simple structure for this article, it also comes with certain limitations—e.g., the range or depth of some of the discussed examples of tranquility extends beyond the category in which they are placed. The categories should therefore only be considered as a preliminary way of mapping and grouping together different examples of tranquil experiences in the hope of achieving some overview of this complex literature. Finally, we propose an exploratory account of tranquility, emphasizing what seems to be shared features among the different experiences of tranquility.

### The body

This category covers experiences wherein the body is calm or tranquil. Noticeable states of bodily tranquility can be found in Indian traditions, e.g., *pratyahara, pranayama*, and *asana* of the Yogis and *passaddhi* of the Buddhists. Here, we focus on one of the most famous examples of bodily tranquility, namely one attained through the yogic posture *shavasana*, i.e., the corpse pose.

In the Yoga Sutras of Patanjali, we are introduced to *ashtanga*, i.e., the “eight limbs of Yoga”: *yama, niyama, asana, pranayama, pratyahara, dharana, dhyana*, and *samadhi* (see Section “The mind” for details). The third limb, *asana*, designates a steady, comfortable position, allowing meditative practice (Satchidananda, 2019, p. 117; YS 2.46). While many today, perhaps especially in Western countries, recognize Yoga as a system of often challenging gymnastic postures, the aim of traditional Yoga was, as already noted, to still the mind, i.e., *nirodha* (YS 1.2, 2.29; Satchidananda, 2019, p. xi). Therefore, some basic seated postures were meant to calm and stabilize the body for meditative purposes in the traditional Yoga of Patanjali. *Padmasana* (the lotus pose) is the most famous meditation pose in Yoga. In medieval times, the Hatha Yoga tradition bloomed with a further exploration of *asanas* [Feuerstein, 2008, pp. 29–31; see Hatha Yoga Pradipika (Akers, 2002)], and since then new postures have been introduced to the world of Yoga (Mallinson, 2017).

In *shavasana*, the practitioner performs a set of postures in a specific routine, which varies depending on the school of Yoga, and then lies down on the floor, relaxing all muscles from head to toes, feet slightly apart, and palms facing upward. The initial set of postures represents the cycle of life, and the final posture, lying down flat on the floor, resembles a corpse. In this symbolic death, the body is relaxed, and this helps to calm the mind [Hatha Yoga Pradipika 1.32 (Akers, 2002, p. 14)]. In the words of the famous Yogi Iyengar (2015, p. 351):

In this asana the object is to imitate a corpse. Once life has departed, the body remains still and no movements are possible. By remaining motionless for some time and keeping the mind still while you are fully conscious, you learn to relax. This conscious relaxation invigorates and refreshes both body and mind. But it is much harder to keep the mind than the body still. Therefore, this apparently easy posture is one of the most difficult to master.

The experience of tranquility is here anchored in the body, which is stilled, relaxing on the floor. Thus, in *shavasana*, one may experience bodily tranquility without experiencing a calm observance of emotions or mind. As emphasized in the quote above, *shavasana* is a practice, whose goal extends beyond calming merely the body.

### Emotions

This broad category covers many concepts for experiences in which emotions are regulated, balanced, or stilled. Most experiences of this category can be subsumed under the notions of emotional equilibrium or equanimity. Some examples of historical concepts of emotional tranquilities are *apatheia* of the stoics, *ataraxia* of the stoics, skeptics, and epicureans, *metriopatheia* by Aristotle, Crantor, and Augustine, *vairagya* and *pratyahara* in Yoga, and *passaddhi* and *upekkha* in Buddhism. Here, we describe *upekkha* (often translated “equanimity” or “even-mindedness”) as found in the Pali-Canon and its role in Theravada Buddhism, and we briefly compare *upekkha* to *apatheia* and *ataraxia* from stoicism.

The first and central teaching of the Buddha was *The Four Noble Truths*. Here, we are told that suffering (*dukkha*) exists, the cause of suffering, the end of suffering, and the path that leads to the end of suffering (i.e., *The Noble Eightfold Path*) [Samyutta Nikaya 56.11 (Bodhi, 2000); Majjhima Nikaya 141 (Nyanamoli and Bodhi, 1995)]. When one follows the *dhamma* (the teachings of the Buddha) through *The Noble Eightfold Path*, one will eventually reach enlightenment (*nibbana*), releasing one from the rebirth of suffering (*samsara*) [Samyutta Nikaya II.15 (Bodhi, 2000)]. According to Buddhist teaching, all phenomena are impermanent (*anicca*), imbued with suffering (*dukkha*), and no-self (*anatta*) (Humphreys, 1969, p. 33; Harvey, 2004, p. 50). From this perspective, we live in ignorance (*avijja*), and our way of being stems from an intuitive, yet illusory feeling of being a self, arising from immediate identification or attachment to our thoughts, emotions (e.g., pleasure or shame), and objects, etc. Since, on this view, no substantial self exists (*anatta*) and everything from emotions to mountains is impermanent (*anicca*), all self-identifications will eventually cause suffering (*dukkha*) and keep the wheels of *samsara* turning.

*Upekkha* is one of the four *brahmavihara*s, i.e., the virtues or meditation practices “which are to be extended boundlessly to all sentient beings” (Bodhi, 2005, p. 154). The other three are: loving-kindness (*metta*), compassion (*karuna*), and altruistic joy (*mudita*) (e.g., Harvey, 2004, p. 209). *Upekkha* is practiced to obtain a calm and balanced state of mind, i.e., a sort of equanimity characterized by emotional detachment, enabling the practitioner to remain neutral and not to react with craving or aversion to whatever occurs (Gowans, 2013, p. 439). Following the Buddhist teaching, the person mastering *upekkha* resists self-identification (i.e., any attachment to self-image, emotions, possessions, etc.) and responds emotionally neutrally to fortune as well as misfortune, thereby preventing suffering [Majjhima Nikaya 54 (Nyanamoli and Bodhi, 1995); see also Anguttara Nikaya 3.65 (Bodhi, 2005, pp. 88–91)]. According to the renowned Buddhist scholar Bhikkhu Bodhi, *upekkha* is perfected through the practice of the other three *brahmavihara*s, and therefore *upekkha* should not be regarded as a disconnection from or disinterest in other people. *Upekkha* is related to the yogic concept of *vairagya* (often translated “detachment,” “dispassion,” or “renunciation”), which designates stages of states in which one is increasingly free from any attachment. In the *Yoga Sutras* of Patanjali, *vairagya* is key to stilling the mind (YS 1.12).

We turn now to the Greek concepts of *apatheia* and *ataraxia*, which, in our view, designate experiences of emotional tranquility that resemble *upekkha.* The meaning of *apatheia* and *ataraxia* differs among the Hellenistic schools (Sorabji, 2000, p. 195f.), and our description of these concepts concerns their role in stoicism only. According to the stoics, virtue is the only good (e.g., Inwood, 2017, p. 78), and living a virtuous life amounts to living a life in agreement with one’s true nature and the universal nature, which, in stoic philosophy, is one and the same. In this context, they emphasize the importance of *apatheia* [Graver, 2007, p. 81; see also Seneca’s *De Tranquillitate Animi*, 2.1–6 (Anderson, 2015)], which designates a calm state of mind where one is not subjugated to one’s passions or prone to acting without deliberation (*propeteia*) (Salles, 2007, p. 249). Dating back to antiquity, views differ as to whether *apatheia* should be understood narrowly as an emotionless state (*apatheia* literally means “absence of passions”) or more broadly as a state of equanimity in which one’s emotions are rational and appropriate to their object—see also the stoic concept of *eupatheiai*, i.e., “good passions” (Frede, 1986; Long, 2002, p. 244; Graver, 2007).

*Ataraxia*, a related concept also used by stoics, literally means “absence of disturbance,” and the stoics conceived *ataraxia* as an imperturbable state related to *apatheia* (Striker, 1990, p. 100f.). In the Hellenistic schools, *ataraxia* was neither a goal in itself nor a constituent of the highest good (i.e., a virtuous life) but rather a consequence of it [Seneca’s *De Vita Beata* 15.2 (Anderson, 2015)]. Although there are obvious similarities between *upekkha*, *apatheia*, and *ataraxia*, there are also differences, e.g., in terms of these tranquil experiences’ relation to the overall goal: *upekkha* is a *constituent* part of the path to prevent suffering, whereas *apatheia* and *ataraxia* are *consequences* of living a virtuous life. In our view, *upekkha*, *apatheia*, and *ataraxia* all designate experiences of tranquility in which emotions are stilled but without necessarily involving a stilled body (as in, e.g., *shavasana*) or a calm observation of the mind.

### The mind

In this category, we explore tranquility of the mind. Here, we describe two kinds of tranquility of the mind, which can be categorized as ‘‘focused awareness’’ and ‘‘open awareness,’’ respectively. To illustrate, we describe *dhyana* meditation of the yogis (exemplifying focused awareness)—*dhyana* is also important in Buddhism (in Mahayana traditions known as *chan* and *zen*, and as *jhana* in Theravada)—and *sati* (‘‘mindfulness’’) of the Theravada Buddhist tradition (exemplifying open awareness).^2^

Recall *ashtanga*, i.e., the eight limbs of Yoga. Only after the yogi has learned to obey the ethical rules (*yama*), internalized these ethical rules as habits (*niyama*), mastered steady and comfortable positions of the body (*asana*), learned to control the breath and energy of the body (*pranayama*), and withdrawn from the senses (*pratyahara*) is the yogi ready for the three final limbs (*samyama*): *dharana, dhyana*, and *samadhi*. These can be regarded as a progressive, three-step meditation practice, leading to enlightenment. *Dharana* (YS 3.1) is a concentration practice in which one binds the attention to one specific object (e.g., the breath, a mantra, or chakra). When the yogi notices that the mind has wandered off (e.g., started thinking), the practice of *dharana* consists in continuously redirecting the attention back to the chosen object. Mastering this, the yogi may slide into *dhyana* (YS 3.2). In this meditative state, the mind completely ceases to wander off, allowing the object of mediation—whatever it may be—to clearly and steadily stand forth. Finally, the yogi is ready to enter the different levels of the absorptive meditative state of *samadhi* (see Section “Mysticism” for details). *Dhyana* is an example of perfected focused awareness, which represents one kind of tranquility of the mind. The Buddhist *samatha* (calm meditation) is like *dharana* with its one-pointed focus. In Theravada Buddhism, both *samatha* and *vipassana* (insight meditation) is needed to achieve true understanding of the nature of reality, i.e., wisdom (*prajna*) and liberation (*nirvana/nibbana*).

Open awareness represents another kind of tranquility of the mind. Contrary to the controlled meditative practice of *dhyana*, *sati* is a matter of a balanced, non-identifying observation. In the *Satipatthana Sutta* of the Pali-Canon, we are told that the person practicing *sati* contemplates the body as body, feeling as feeling, mind as mind, mind-objects as mind-objects in their appearing or vanishing states [Majjhima Nikaya 10 (Nyanamoli and Bodhi, 1995, pp. 145–155)]. Basically, this means that whatever appears in meditation (e.g., thoughts, emotions, or external sounds) is experienced without reaction, i.e., without grabbing on to them due to craving or pushing them away due to aversion. Thus, *sati*, contrary to *dharana*, does not involve binding and redirecting one’s attention to a chosen object but instead in fostering an alert and attentive (mindful) state. By practicing *sati*, one cultivates, as Analayo (2006, pp. 263–264) put it, “bare and equanimous receptivity, combined with an alert, broad, and open state of mind.” Although the body may not be stilled (as in *shavasana*), and emotions and thoughts may not be quieted, the practitioner in *sati* notices everything from within a calm and tranquil state of receptive presence or equanimity, which is characterized by an open, balanced, non-identifying attitude toward whatever appears in consciousness. *Sati* differs from *upekkha* or *ataraxia*, which are focused on emotional imperturbability, whereas *sati* rests on a meta-cognitive capacity of noticing and letting-be of every—pleasant or unpleasant—event.

### Mysticism

Mystical experiences cover a wide range of states (including visions, trances, and ruptures), but here we focus solely on what often is considered the most significant type of mystical experience (e.g., Otto, 1931; Stace, 1961), namely *unio mystica.*^3^ The interpretation of *unio mystica* varies, depending on the context in which it occurs [e.g., the One (Plotinus), the Godhead/divinitas (Eckhart), *shunyata*, *nirvana*/*nibbana* (Buddhism), and *moksha*/*mukti*/*kaivalya* (Indian philosophy, Hinduism, etc.)], but its experiential nucleus has by some authors been proposed to be the same, i.e., an ineffable, boundless sense of undifferentiated oneness or unity with the Absolute (Stace, 1961; Parnas and Henriksen, 2016).^4^ Otto (1931, p. 39) famously distinguished between two types of mystical union: the inward way (“mysticism of *introspection*”) and the outward way (“mysticism of *unifying vision*”). In the first, “The secret way leads *inward*” (Otto, 1931, p. 40), i.e., it implies a complete withdrawal from everything outward and a retreat into the depths of the mind, culminating in a non-sensuous, mystical experience of union. The outward way, by contrast, “knows nothing of “inwardness” (…) It looks upon the world of things in its multiplicity” (Otto, 1931, p. 42), culminating in seeing unity or oneness shine through everything in the sensory field. Otto’s distinction was later echoed in Stace’s (1961, p. 61f.) division between introvertive (“looks inward into the mind”) and extrovertive (“looks outward through the senses”) mysticism. Using this classic distinction, we describe two kinds of mystical experience: *samadhi* in Indian philosophy (exemplifying the inward way) and the *One Mind* of Huang Po, a ninth-century Chinese master of Chan (Zen) Buddhism (exemplifying the outward way).

The practices that lead to *samadhi* and its interpretation vary among the Indian schools. We focus here on the final and highest stage of *samadhi*, i.e., *asamprajnata samadhi*, as described in the Yoga Sutras of Patanjali. As noted above (see Section “The mind”), *samadhi* is the eighth and final limb of Yoga, expressing progressively deep meditative stages of absorption, ecstasy, and bliss [YS 2.28–29; see Feuerstein (2008, pp. 208, 216, 398)]. After enduring and dedicated practice, following *ashtanga*, the yogi may eventually reach *asamprajnata samadhi*. In this final stage of *samadhi*, which is devoid of any object of meditation, the yogi realizes his or her true self (YS 1.16, 1.18), which means that the yogi’s consciousness is unified with the absolute or cosmic consciousness. In this ultimate stage of *samadhi*, all duality has ceased, and only pure consciousness remains. Satchidananda describes it as a state “where even the ego feeling is not present and the seeds of past impressions are rendered harmless. In that state, only consciousness is there and nothing else. Once that is achieved, the individual is completely liberated and there is no more coming into the world and getting tossed” (Satchidananda, 2019, p. 33). And further, “in Samadhi, you don’t even know (that you are in meditation). You are not there to know it because you are that (…) there is neither the object nor the meditator. There is no feeling of “I am meditating on that” (…) you and God become one. That’s Samadhi” (Satchidananda, 2019, p. 165).^5^ *Asamprajnata samadhi* exemplifies a state of mystical tranquility, reached by “the inward way.” Contrary to the tranquilities of the body, emotions, and the mind, which we presented in the previous sections, everything external is shut off and all bodily, emotional, and mind-related dynamics are completely stilled or quieted in *asamprajnata samadhi*, leaving nothing but a tranquil experience of pure consciousness. It is an experience of absolute emptiness and fullness at once. Notably, experiences of mystical union, reached through the inward way, are also described in other mystical texts and traditions (e.g., in Vedantic texts as opposed to the Yogic one, we cited before, but also in, e.g., Jewish, Christian, and Islamic mysticism).

Finally, we consider Huang Po’s description of the *One Mind* as an example of “the outward way.” Huang Po distinguishes between what he calls the conceptual mind and the *One Mind*, which is the Buddha nature of all sentient beings, i.e., everything is one. According to Huang Po, one cannot grasp the true Buddha nature through conceptualization. If one reaches for the truth, using the conceptual mind, one will, as he put, be “cut off and (…) find nowhere to enter” [1.9 (Blofeld, 1958)]. He continues, “there is only one reality, neither to be realized nor attained. To say “I am able to realize something” or “I am able to attain something” is to place yourself among the arrogant (…) there is just a mysterious tacit understanding and no more” [1.17 (Blofeld, 1958)]. Huang Po described the experience of the Buddha nature as a state of being detached from conceptualization and form [1.5–6 (Blofeld, 1958)], where speech is silenced, and all mental movement is stilled [2.17; see also 2.42 (Blofeld, 1958)]. He sums it up as follows, “our original Buddha-Nature (…) is void, omnipresent, silent, pure; it is glorious and mysterious peaceful joy—and that is all” [1.8 (Blofeld, 1958)].^6^

Like *asamprajnata samadhi*, Huang Po’s *One Mind* exemplifies a state of mystical tranquility. Contrary to *asamprajnata samadhi*, however, Huang Po’s *One Mind* requires neither a detachment from one’s immersion in the world [1.6; see also 2.42 (Blofeld, 1958)] nor a progressive, inward search through still deeper stages of meditation through which all bodily, emotional, and mind-related phenomena eventually are stilled, leaving the mind completely empty and receptive of the mystical union. Rather Huang Po, whose teaching today is followed by the Rinzai-Zen community, believed in a sudden realization, sometimes within a second, perhaps provoked by hearing the teaching [1.6 (Blofeld, 1958)] or by receiving a blow to the head from one’s teacher [2.28 (Blofeld, 1958)]. This is of course not to overlook or underestimate the importance of training and preparing the mind through meditation about which Huang Po, however, did not offer much detail (Blofeld, 1958, p. 19). Huang Po’s *One Mind* articulates an experience of mystical union, i.e., seeing one in all. In *One Mind*, only the conceptual mind is stilled, leaving nothing but a tranquil, peaceful joy.

## An exploratory account of tranquility

The described tranquil experiences include a broad selection of experiences that in many ways differ from each other, and we can clearly see their respective cultural or religious imprints. Despite their differences, they seem to share some intriguing experiential features. To varying degrees, they all entail a sense of presence and inner peace, sometimes associated with pleromatic sensations such as warmth, bliss, flow, and release of tension. Apart from these features, which mainly concern the *content* or *quality* of tranquility, experiences of tranquility seem also to share, again in varying degrees, a two-sided *structural* feature of detachment and absorption.

Detachment has been a key concept in several schools of thought in East and West, reflected in concepts such as *vairagya* in Yoga and *Abgeschiedenheit* in the works of Meister Eckhart. Etymologically, “to detach” (from old French, *destachier*; *des “*apart” and *attachier* “attach or connect”) means “to untie” or “to disconnect.” Detachment comes in different degrees, ranging from a limited kind that concerns only one domain (e.g., the disconnection from passions in *apatheia*) to an unlimited kind in which everything eventually is obliterated from consciousness (e.g., in *asamprajnata samadhi*). In the Eastern schools, detachment is regarded as a disconnection from or discontinuation of the ongoing self-identification with bodily sensations, emotions, or thoughts, etc. Indeed, the eight limbs of Yoga (*ashtanga*) or the Buddhist meditative practices can all be interpreted as gradually intensifying practices to soften, loosen, and eventually to let go of any self-identification, which is considered the central obstacle for spiritual enlightenment in these traditions. For example, dedicating the fruits of one’s labor to God instead of taking pride in it (YS 3.1; cf. *bhakti yoga* of the Bhagavad Gita) or, in meditation, redirecting one’s attention to the chosen object (*dharana*) instead of being immersed and invested in whatever thoughts or emotions pop up is basically to practice this kind of detachment (*vairagya*). The more absolute this detachment is, the more the meditator is emptied of all self-bound phenomena. Finally, letting go of any self-identification amounts to breaking through the self-illusion in *samadhi* or *nirvana/nibbana*. The basic idea that the self must be destroyed for the practitioner to become receptive of the mystical union is also found in other traditions. In Sufism, the concept of *fana* (Arab *faniya*, “to pass away,” “to perish”) designates the annihilation of the self (*nafs*) that separates the human being from God—as Wilcox (2011, p. 95) put it, “the passing away of the self is thus the essential pre-requisite to the survival (*baqa*) of the selfless divine qualities placed in man by God.” In Christian theology, the concept of *kenosis* denotes the emptying of the self. In Christian mysticism, this theme was particularly emphasized in the works of Meister Eckhart, who devoted a thesis to the subject of detachment. Here, Eckhart (2009, pp. 556–575) “quotes” St. Augustine—though the quote is not actually found in St. Augustine’s works—for stating, “The soul has a secret entrance to the divine nature, when all things become nothing for it” (Eckhart, 2009, p. 573). According to Eckhart, “this entrance is nothing but pure detachment” (Eckhart, 2009), i.e., only by liberating oneself from all needs, strivings, and desires can the mind become completely empty, unmoved by whatever occurs, “rest on absolutely nothing” (Eckhart, 2009, p. 572), and thus be “receptive of nothing but God” (Eckhart, 2009, p. 567f.).

In sum, the experiences of tranquility exhibit, to varying degrees, the structural character of detachment—from the disconnection of the incessant self-involvement with our bodily sensations, emotions, or thoughts to the complete self-annihilation in experiences of mystical union. These different degrees and perhaps even different kinds of detachment may bring about various experiences on both the so-called “self-pole” and “world-pole” of experience—e.g., on the “self-pole,” we find descriptions of “pure experience” (Zen), “witness consciousness” [Advaita Vedanta (Gupta, 1998) and Buddhism (Albahari, 2009)], and “the white light of the self” [Ramana Maharshi (Mudaliar, 1965)], whereas, on the world-pole, we find descriptions of experiencing objects as instantiations of oneness in the unifying vision.

Yet, the experiences of tranquility are, in our view, not adequately described as only involving detachment, which, briefly put, refers to an inhibition, discontinuation, or disconnection from something that usually is present. By contrast, the detachment that characterizes tranquil experiences seems simultaneously to imply some degree of absorption into another kind of awareness. Etymologically, “absorption” (Latin *absorbere*, from *ab* “off, away from” and *sorbere* “suck in”) means to be “swallowed up” or “taking in by” something. In research on hypnosis, absorption has been defined both as a personality *trait*, designating a propensity or readiness for experiences of profound involvement in something (e.g., Tellegen and Atkinson, 1974), and as an experiential *state* in which one is totally immersed and directing all of one’s resources to a specific attentional object (Kumar et al., 1996). Interestingly, absorptive states have here been described as involving “a heightened sense of reality of the attentional object, imperviousness to distracting events, and an altered sense of reality in general, including an empathically altered sense of self” (Kumar et al., 1996, p. 232). Our use of the concept of absorption bears similarity to this description of absorptive states. Yet, where absorptive states in hypnosis are said to involve an altered sense of reality *in general*, we suggest that this is not the case for *all* the forms of absorption that are at stake in experiences of tranquility. For example, detaching from emotions in *upekkha* or passions in *apatheia* involves absorption into a calm state of equanimity. In meditational practices such as *dharana* and *dhyana*, the meditator detaches from the ordinary and immediate self-identification and self-involvement with bodily sensations, emotions, and thoughts as they ceaselessly appear, disappear, and reappear in consciousness. The constant redirection of awareness to the chosen object in *dharana* or the undisturbed awareness of the chosen object in *dhyana* involves absorption into a kind of focused awareness. In *sati*, the meditator notices whatever pops up in the mind but without doing anything about it, except noticing it. Here, too, the meditator detaches herself from the usually incessant self-involvement and preoccupation with bodily sensations, emotions, and thoughts and is instead absorbed into a kind of open awareness. In *sati*, we may say, using Fasching’s description, that the meditator becomes aware of “the self-presence of experiencing itself (…) become conscious of consciousness itself (which usually remains “hidden” behind what it is conscious of)” (Fasching, 2008, p. 464). Finally, at the level of mysticism, the experience of *One Mind* involves detachment from our ordinary mode of being and sensing (i.e., detachment from the “conceptual mind” in Huang Po’s terms) and, simultaneously, absorption into the experience of oneness (the Buddha nature) as it unfolds in the unifying vision. The most absolute kind of absorption co-occurs with the most absolute kind of detachment. It is found in experiences of mystical union that are reached through the inward way. Here, everything is obliterated from the mind, and only the experience of mystical union is present. In our view, it is only at the level of mysticism that the absorptive states genuinely involve an altered sense of reality, including an altered sense of self.

Finally, our description of tranquility would be incomplete if we failed to mention that to reach most of the described tranquil experiences, it is, across traditions such as stoicism or yoga, Buddhism or Christianity, considered a prerequisite to live an ethical-spiritual life in accordance with the culturally or spiritually defined virtues and rules; or, as bluntly stated in the Book of Isaiah, “there is no peace for the wicked” (48:22). Although living an ethical life usually is considered a prerequisite for experiencing tranquility, ethical living is not itself a tranquil experience. Therefore, an exploration of the ethical dimension of tranquility, though important, is beyond the scope of our study.

## Concluding remarks

In this study, we have shown that experiences of tranquility come in many different shapes and colors, attesting to the complexity of the phenomenon. By exploring experiences of tranquility across Eastern and Western traditions, we argued that these experiences share certain core features both in terms of their experiential content or quality (i.e., a sense of presence and inner peace) and structure (i.e., detachment and absorption). However, even if one concedes that these core experiential features indeed characterize tranquility, one cannot conclude that they necessarily define it. A definition, specifying the essence of tranquility, requires drawing a conceptual boundary between tranquility and seemingly related phenomena, which also involve some degree of presence, peace, absorption, or detachment. Exploring certain absorptive states of artistic (Høffding, 2019), esthetic (Legrand and Ravn, 2009), or athletic peak performance (Privette, 1983) could be relevant candidates for such a comparative endeavor. If a clear boundary cannot be drawn between tranquility and other related phenomena, then the definition would either fall short or, alternatively, one must grant that these phenomena too entail an element of tranquility. Such analyses, however, lie beyond the scope of our study. Consequently, we do not propose a definition of tranquility but point instead to shared experiential features that may be useful for further research on tranquility.

When exploring experiences of tranquility across different cultures and searching for core features of such experiences, one is inevitably confronted by the question of whether such experiences possess a universal nature or if they instead are socially or culturally constructed. This debate is prominent in mysticism research, where the controversy boils down to a distinction between two positions, i.e., the perennials view and the constructivist view. The perennials view argues for a universal nature of mystical experiences that is discernable across cultures and traditions. This view has been advocated by scholars like William James, Aldous Huxley, and Walter T. Stace (Stace, 1961). The constructivist view, however, criticizes the perennials view for being epistemologically naïve, ignoring constitutive aspects of sociocultural, religious, and historical contexts on mystical experiences. Steven T. Katz, one of the most influential advocates of the constructivist view, argues that mystical experiences are radically different, and consequently he emphasizes the need for epistemological pluralism (Katz, 1978). However, with new insights and hermeneutic rigor, which was introduced in the wake of the constructivist’s criticism of the early perennialists, we have witnessed something like a rehabilitation of the perennials view (Forman, 1999). Research on shared core features of mystical experiences has been juxtaposed with analyses of sociocultural, religious, and historical contexts in determining the mystical experiences’ variability (Smith, 1987). In our view, such an approach of what could be labeled “moderate perennialism” seems appropriate for studying experiences of tranquility, which, in our view, both share certain experiential features and remain influenced by the culture and tradition in which they are embedded.

In the absence of reviews on experiences of tranquility and lack of consensus about the concept’s meaning, we considered a theoretical, explorative study adequate for the purpose of keying in on the experiential nature of tranquility. This approach allowed us to explore and synthesize insights into experiences of tranquility from many influential traditions, spanning continents and millennia. Yet, our analyses are constrained by our knowledge of such traditions and language barriers, and we may have overlooked nuances between the concepts. These limitations notwithstanding, the study has provided insights into the experiential nature of tranquility, its content and structure, and these insights may serve as a vehicle for further research, not only narrowly on tranquility, but also more broadly on other disciplines and research areas on human subjectivity such as consciousness studies, mysticism and religious studies, meditation, mental health, mental disorders, psychotherapy, and rehabilitation, etc. In a time of global health crisis, it is important to remember that experiential tranquility in many cases can be reached within, and that tapping into its deep well may not only have benefits for ourselves but also for those around us.

## Author contributions

VRC wrote the first draft of the manuscript, which was revised by MGH and BŠ. All authors jointly formulated the study’s purpose and approved the final version of the manuscript.

## Footnotes

1 Our reading of Patanjali’s Yoga Sutras is based on translations and commentaries by Karambelkar (2012) and Satchidananda (2019).

2 Since Western mindfulness is strongly based upon Buddhist meditative practices (Kabat-Zinn, 2011), we do not explore potential differences between Western concepts of mindfulness, and say, *sati* of Theravada Buddhism.

3 Other mystical experiences include *kaivalya* of various Indian traditions, *moksha* of Hinduism, *nibbana* of Buddhism, Meister Eckhart’s *Godhead*, *hesychia* of Eastern Orthodox Hesychasm, the *bardo*-state of Tibetan Buddhism, *bitul ha-yesh* of Jewish Chabad philosophy, the Daoist state of *miejin ding*, the Zen Buddhist states of *kenshô* and *satori*, and *wagd* of Sufism.

4 Later, we address the role of culture in mystical experiences as we discuss the so-called perennials and constructivist views on the interpretation of experiences of unio mystica.

5 The sentence “You are not there to know it because you are that” might seem unfinished. It is not. The phrase “you are that” refers to a core thought of Vedantic philosophy, based on the Sanskrit mantra *Tat Tvam Asi* (“thou art that”) from the famous Chandogya Upanishad (e.g., Myers, 1993). The phrase refers to the unity of the individual self (*Atman*) and God (*Brahman* or the Absolute).

6 Notably, similar reports of sudden realization of oneness shining through all diversity can also be found in other traditions, e.g., in Christian mystics such as Meister Eckhart or Jakob Boehme. In a famous passage from *The Aurora*, Boehme stated, “In this Light my Spirit suddenly saw through all, and *in* and *by* all the Creatures, even in Herbs and Grass, it knew God” (Boehme, 1764, p. 184).
